The article "lncRNA Gm15290 promotes cell proliferation and invasion in lung cancer through directly interacting with and suppressing the tumor suppressor miR-615-5p" was published in 2018. Journal: Biosci Rep.

# lncRNA Gm15290 promotes cell proliferation and invasion in lung cancer through directly interacting with and suppressing the tumor suppressor *miR-615-5p*

**DOI:** 10.1042/BSR20181150

**Published:** 2018-10-31

**Authors:** Yu Dong, Xiaoying Huo, Ruiying Sun, Zhiyan Liu, Miaoyi Huang, Shuanying Yang

**Affiliations:** 1 Department of Respiratory Medicine, Xi’an Central Hospital, Xi’an, China; 2 Department of Respiration Medicine, the Second Affiliated Hospital of Xi’an Jiaotong University, Xi’an, China; 3 Department of Respiratory Medicine, Fourth Hospital of Xi’an, Xi’an, China

**Keywords:** cell proliferation and invasion, lncRNA Gm15290, miR-615-5p, non-small cell lung cancer, RNA interaction

## Abstract

Long non-coding RNAs (lncRNAs) have been involved in occurrence and progression of multiple cancers. In the present study, we investigated the role of lncRNA Gm15290 in the proliferation and invasion of non-small cell lung cancer (NSCLC) cells. First, we found that lncRNA Gm15290 was markedly up-regulated in tumor tissues from NSCLC patients and NSCLC cell lines, compared with adjacent normal tissues and normal lung cell line HBE respectively. Then, different concentrations of pcDNA-Gm15290 expression vector and Gm15290 siRNA were respectively transfected into A549 NSCLC cells. Our results showed that overexpression of Gm15290 significantly increased the proliferation and invasion of A549 cells and suppressed cell apoptosis. Knockdown of Gm15290 suppressed A549 cell proliferation and invasion and promoted cell apoptosis. Subsequently, we explored the underlying mechanism through which Gm15290 promoted cell proliferation and invasion. The output of RNA hybrid bioinformatic tool revealed that Gm15290 potentially interacted with tumor suppressor *miR-615-5p* which displayed an opposite expression pattern in the cell lines and a strong negative correlation with the levels of Gm15290 in NSCLC patients (r^2^ = 0.9677, *P*<0.0001). The results of RNA pull-down assays confirmed that Gm15290 directly bound with *miR-615-5p*. Gm15290 negatively regulated the expression of *miR-615-5p* and increased the protein levels of *miR-615-5p* target genes, including *IGF2, AKT2*, and *SHMT2*. Moreover, *miR-615-5p* mimic could antagonize the promoting effect of Gm15290 on cell proliferation and invasion.

## Introduction

Lung cancer has become the leading cause of cancer death in China. Non-small cell lung cancers (NSCLC), including squamous cell carcinoma, adenocarcinoma, and large cell carcinoma, account for more than 80% of lung cancer cases [1]. In contrast with small cell lung cancer cells, the growth and division of NSCLC cells are much quicker, and their invasion to adjacent tissues and distant metastasis are much earlier [2,3]. More than half of the non-small cell lung tumors are diagnosed at advanced stages, so that the 5-year survival rate of NSCLC patients is lower than 15% [4–6]. The pathogenesis of NSCLC is not yet fully understood. Therefore, it is urgent to unearth reliable diagnostic and therapeutic targets for NSCLC.

The article "lncRNA Gm15290 promotes cell proliferation and invasion in lung cancer through directly interacting with and suppressing the tumor suppressor miR-615-5p" was published in 2018. Journal: Biosci Rep.

Long non-coding RNAs (lncRNAs) are non-protein coding RNA transcripts longer than 200 nts [7]. During the past decade, lncRNAs have become a category of ncRNAs with the largest number and the most abundant regulatory manners [8,9]. They played important roles in fine regulation of gene expression by directly or indirectly interacting with DNAs, mRNAs, proteins, and other categories of ncRNAs [10,11]. Some recent studies on transcriptomes and ncRNA expression profiles revealed that lncRNAs have been involved in tumor growth, invasion, metastasis, and drug resistance of multiple cancers including NSCLC, and that they regulated proto-oncogenes or tumor suppressor genes in many different ways [12–15]. Take lncRNA HOX transcript antisense RNA (HOTAIR) as an example, this famous lncRNA is up-regulated in the NSCLC tissue compared with the adjacent normal tissue, elevated expression of which has been demonstrated to be correlated with invasion, metastasis, and poor survival in patients with NSCLC [16]. HOTAIR could shift polycomb-group protein 2-mediated gene repression from tumorigenic genes to tumor-suppressive genes [17], it could interact with E3 ubiquitin ligases and their corresponding substrates through specific RNA binding domains to proteolyse oncogenes Ataxin-1 and Snurportin-1 [18], and it also could interact with several miRNAs that played positive or negative roles in tumor development [19,20]. Some other lncRNAs also played important roles in tumor development and drug resistance through interacting with coding genes or ncRNAs, such as UCA1 and AK126698 [21,22]. More and more lncRNAs are being found and their roles in the progression of NSCLC are to be revealed.

*miR-615-5p* was transcribed from the host gene homeobox C4 on Chromosome 12 in human [23]. Several studies have revealed the tumor suppressive role of *miR-615-5p* in some parenchymatous tumors, including hepatocellular carcinoma and pancreatic ductal adenocarcinoma [23,24]. It was demonstrated that *miR-615-5p* could directly target multiple oncogenes, suppress their expression, and inhibit their mediated tumor growth and metastasis. In the present study, we explored the role of Gm15290, a quite newly discovered lncRNA, in the proliferation and invasion of NSCLC cells. The levels of Gm15290, in the NSCLC tissues compared with adjacent normal tissues and in the human normal lung epithelial cell line compared with NSCLC cell lines, were detected. Then, different concentrations of pcDNA-Gm15290 expression vector and Gm15290 siRNA were respectively transfected into A549 NSCLC cells to uncover its exact role in cell proliferation and invasion. Moreover, we found that the role of Gm15290 in NSCLC progression was related to *miR-615-5p*, a previously identified tumor suppressor miRNA.

The article "lncRNA Gm15290 promotes cell proliferation and invasion in lung cancer through directly interacting with and suppressing the tumor suppressor miR-615-5p" was published in 2018. Journal: Biosci Rep.

## Materials and methods

### Ethics statement and specimens

The study was approved by the Ethical Committee of the Second Affiliated Hospital of Xi’an Jiaotong University, and all the subjects gave written informed consent to participate in the study. The study enrolled 30 NSCLC patients aged (50 ± 10.5) years, with 15 males and 15 females. Carcinoma tissues and matched adjacent normal tissues were sampled from each subject by minimal invasive surgery. The tissue specimens were store at −80°C for subsequent use.

### Cell culture

HBE normal lung epithelial cell line and three NSCLC cell lines, including SK-MES-1, A549, and NCI-H460, were purchased from Cell Center of Xi’an Jiaotong University (Xi’an, China). The cells were taken from liquid nitrogen and then thawed in 37°C water bath. HBE, SK-MES-1, and A549 cells were grown in DMEM (Invitrogen, Carlsbad, CA) containing 4.5 g/l glucose, 4 mmol/l L-glutamin supplemented with 10% FBS (Invitrogen). NCI-H460 cells were grown in 1640 medium (Invitrogen) containing 4.5 g/l glucose and 4 mmol/l L-glutamin, supplemented with 10% FBS. The cells were incubated in a humidified incubator with an atmosphere of 95% air-5% CO_2_ at 37°C.

### Transfection

The pcDNA-Gm15290 expression vector was constructed by GenScript Company (Nanjing, China). Specific siRNA against Gm15290 and single-strand *miR-615-5p* mimic were designed, synthesized, and validated effective by Ribobio Company (Guangzhou, China). For transfection, the cells were seeded into six-well plates at the density of 10^5^/cm^2^. On reaching 70% of confluence, the pcDNA-Gm15290, Gm15290 siRNA, and *miR-615-5p* mimic were individually transfected or co-transfected into the A549 cells with Lipofectamine 3000 (Invitrogen) according to the manufacturer’s instructions.

### Cell proliferation, apoptosis, and invasion analysis

Cell proliferation was evaluated using the Cell Counting Kit-8 (CCK-8; Sigma, St. Louis, MO) assay. The cells were incubated for 24, 48, and 72 h before adding 200 μl of CCK-8 reagent to each well and incubated at 37°C for 2 h. Cell proliferation was measured by absorbance at 450 nm wavelength using a microplate reader (Bio-Rad, Hercules, CA).

Cell apoptosis was detected with a PI/AnnexinV Cell Apoptosis Detection Kit (Sigma). Following transfection for 48 h, 10^6^ cells (in 1 ml medium) were washed with cold PBS and centrifugated at 1000 rpm for 5 min. The cells were resuspended by 10 μl of AnnexinV-FITC solution that followed by a 15-min incubation on ice. Then, the cells were transferred into the detection tube with 500 μl of PBS and 5 μl of PI solution. After another 2 min, the cells were analyzed by a flow cytometry (Bio-Rad). The percentage of early apoptotic cells (AnnexinV^+^PI^−^) was calculated.

The article "lncRNA Gm15290 promotes cell proliferation and invasion in lung cancer through directly interacting with and suppressing the tumor suppressor miR-615-5p" was published in 2018. Journal: Biosci Rep.

Cell invasion was detected with the transwell cell invasion assay. Briefly, the assay was performed with a Matrigel (Sigma) coated on the upper surface of the transwell chamber (Corning, Lowell, MA). The cells that had migrated through the membrane were fixed with methanol and stained with crystal violet. Photographs of three randomly selected fields of the stained cells were taken, and cell numbers were counted by a Countess Automatic Cell Counter (Invitrogen).

### Real-time quantitative PCR

Total RNA was isolated using TRIzol reagent (Invitrogen). Real-time qPCR reactions were carried out in a 25-μl system using SYBR Premix Ex Taq (TaKaRa), 0.4 mM of each primer, and 200 ng of cDNA template. Specific primers for Gm15290, 18S RNA mature, *miR-615-5p*, and U6 RNA were designed and synthesized by Ribobio Company (Guangzhou, China). Each individual sample was run in triplicate wells. PCR amplification cycles were performed using SYBR Premix Ex Taq II Kit (Invitrogen) and analyzed by iQ^TM^ 5 Multicolor Real-Time PCR Detection System (Bio-Rad). The reactions were initially denatured at 95°C for 2 min, followed by 35 cycles of 95°C for 15 s, and 60°C for 60 s. RNA enrichments were calculated using the 2^−ΔΔ*C*^_T_ method.

### Western blotting

Fifty micrograms of total protein from each sample was separated by 12% SDS/PAGE and electro-transferred onto PVDF membranes (Millipore, Boston, MA) for immunoblotting analysis. The primary antibodies including Anti-IGF2 (1:500, Abcam), Anti-AKT2 (1:500, Abcam), Anti-SHMT2 (1:300, Abcam), and Anti-β-actin (1:800, Abcam) were used to incubated with the membranes at 4°C overnight. After incubation with appropriate Horseradish Peroxidase-conjugated secondary antibodies, the blots were detected using Immobilon ECL Kit (Millipore) in a ChemiDoc XRS Imaging System and analyzed by Quantity One software (Bio-Rad).

### Pull-down assay with biotinylated Gm15290 cDNA probe and Northern blot analysis for the enrichment of *miR-615-5p* bound by Gm15290

The biotinylated DNA probe complementary to Gm15290 and negative control probe were designed and synthesized by Invitrogen and dissolved in 500 μl of binding buffer (0.5 M NaCl, 20 mM Tris-HCl, pH 7.5, and 1 mM EDTA). The probes were incubated with streptavidin-coated magnetic beads (Sigma) at room temperature for 3 h to obtain probe-coated magnetic beads. Cell lysates were incubated with probe-coated beads, and the RNA complexes pulled down were eluted and extracted for the following Northern blot analysis.

The article "lncRNA Gm15290 promotes cell proliferation and invasion in lung cancer through directly interacting with and suppressing the tumor suppressor miR-615-5p" was published in 2018. Journal: Biosci Rep.

The RNA complexes were run on a 15% polyacrylamide-urea gel and transferred to positively charged nylon membranes (Millipore) followed by cross-linking through UV irradiation. The membranes were subjected to hybridization with 3′-digoxigenin-labeled probes overnight at 4°C. The *miR-615-5p* probe and U6 RNA probe were labeled with digoxigenin using a 3′-End Digoxigenin Labeling Kit (Roche). The detection was performed using a Digoxigenin Luminescent Detection Kit (Roche) according to the manufacturer’s instructions.

### Pull-down assay with biotinylated miRNA

A549 cells were transfected with 50 nM of wild type biotinylated *miR-615-5p* or the mutated biotinylated *miR-615-5p* probes. After incubation for 48 h, cells were harvested, washed with cold PBS followed by brief vortex, and incubated in a lysis buffer (20 mM Tris, pH 7.5, 200 mM NaCl, 2.5 mM MgCl2, 0.05% Igepal, 60 U ml 1 Superase-In (Ambion), 1 mM DTT, protease inhibitors (Roche) on ice for 10 min. The lysates were precleared by centrifugation, and 50 μl of the sample was aliquoted for input. The remaining lysates were incubated with M-280 streptavidin magnetic beads (Sigma). To prevent non-specific binding of RNA and protein complexes, the beads were coated with RNase-free BSA and yeast tRNA (both from Sigma). The beads were incubated at 4°C for 3 h, washed twice with ice-cold lysis buffer, three-times with the low salt buffer, and once with the high salt buffer. The RNA complexes pulled down were purified by TRIzol reagent and then applied in the qPCR analysis for lncRNA-Gm15290 enrichment.

### Website references

The targetting relationship between Gm15290 and *miR-615-5p* was calculated by an online server RNA hybrid (http://bibiserv.techfak.uni-bielefeld.de/rnahybrid/).

### Statistical analysis

Values were expressed as means ± S.E.M. obtained from at least three independent experiments. Statistics were calculated by SPSS 22.0. Multiple comparisons were assessed by one-way ANOVA that followed by Dunnett’s tests. The correlation between the levels of Gm15290 and *miR-615-5p* was evaluated by the Pearson correlation coefficient analysis. Differences between groups were considered statistically significant if *P*<0.05.

## Results

### lncRNA Gm15290 was significantly up-regulated in human NSCLC tissues and cell line

Expression of lncRNA Gm15290 in cancerous tissues and matched adjacent normal tissues from 30 NSCLC patients was detected with real-time qPCR. The results showed that Gm15290 was up-regulated to about 3-folds in the cancerous tissue, compared with the adjacent normal tissue (Figure 1A). Then, Gm15290 expression in HBE human normal lung epithelial cell line and three NSCLC cell lines, including SK-MES-1, A549, and NCI-H460 was detected. We found that Gm15290 was increased to more than 5-folds in the NSCLC cell lines (Figure 1B). These data suggest that Gm15290 is likely to play a role in NSCLC progression.

The article "lncRNA Gm15290 promotes cell proliferation and invasion in lung cancer through directly interacting with and suppressing the tumor suppressor miR-615-5p" was published in 2018. Journal: Biosci Rep.

**Figure 1:** lncRNA Gm15290 was up-regulated in human NSCLC tissues and NSCLC cell lines (**A**) Gm15290 was up-regulated in the carcinoma tissues from NSCLC patients compared with matched adjacent normal tissues. Carcinoma tissues and matched adjacent normal tissues were isolated from 30 patients with NSCLC. Total RNA was isolated and Gm15290 expression was detected with qPCR. (**B**) Gm15290 was up-regulated in human NSCLC cell lines. The expression of Gm15290 in HBE human normal lung epithelial cell line and three human NSCLC cell lines, including SK-MES-1, A549, and NCI-H460, was detected with qPCR. **P<0.01 compared with HBE.

### Overexpression of Gm15290 promoted proliferation and invasion and suppressed apoptosis in A549 NSCLC cells

To investigate the role of Gm15290 in the progression of NSCLC, different concentrations of pcDNA-Gm15290 overexpression vector were transfected into A549 cells. The level of Gm15290 was significantly increased by 1 μg/ml of pcDNA-Gm15290 and dramatically increased by 2 and 4 μg/ml of pcDNA-Gm15290 (Figure 2A). The results of CCK-8 assay and transwell cell invasion assay showed that Gm15290 overexpression promoted proliferation and invasion of A549 cells in a dose-dependent manner (Figure 2B,D). Simultaneously, Gm15290 overexpression suppressed apoptosis of A549 cells in a dose-dependent manner (Figure 2C).

**Figure 2:** lncRNA Gm15290 overexpression promoted the proliferation and invasion of A549 NSCLC cells (**A**) The overexpression efficiency of the Gm15290 by the pcDNA-Gm15290 at different concentrations. (**B**) Gm15290 overexpression increased the proliferation of A549 cells in a dose-dependent manner. (**C**) Gm15290 overexpression suppressed the apoptosis of A549 cells in a dose-dependent manner. (**D**) Gm15290 overexpression promoted the invasion of A549 cells in a dose-dependent manner. The pcDNA-Gm15290 expression vector at concentrations of 1, 2, and 4 μg/ml were respectively transfected into A549 cells. After incubation for 48 h, the Gm15290 enrichment was detected with qPCR, cell proliferation was CCK-8 assay, cell apoptosis was detected with flow cytometry, and cell invasion was detected with transwell cell invasion assay. *P<0.05 compared with vector, **P<0.01 compared with vector.

The article "lncRNA Gm15290 promotes cell proliferation and invasion in lung cancer through directly interacting with and suppressing the tumor suppressor miR-615-5p" was published in 2018. Journal: Biosci Rep.

### Knockdown of Gm15290 inhibited proliferation and invasion and increased apoptosis of A549 NSCLC cells

To further investigate the role of Gm15290 in the proliferation and invasion of NSCLC cells, different concentrations of Gm15290 siRNA were transfected into A549 cells. In contrast with the results from Gm15290 overexpression, the level of Gm15290 was significantly decreased by 20 nM of Gm15290 siRNA, and dramatically decreased by 40 and 80 nM of Gm15290 siRNA (Figure 3A). Gm15290 knockdown inhibited proliferation and invasion of A549 cells in a dose-dependent manner (Figure 3B,D). Simultaneously, Gm15290 knockdown promoted apoptosis of A549 cells in a dose-dependent manner (Figure 3C). These data combined with the data from Gm15290 overexpression experiments indicate that Gm15290 positively regulates proliferation and invasion of A549 NSCLC cells and negatively regulates their apoptosis.

**Figure 3:** lncRNA Gm15290 knockdown suppressed the proliferation and invasion of A549 cells (**A**) The knockdown efficiency of the Gm15290 by the Gm15290 siRNA at different concentrations. (**B**) Gm15290 knockdown reduced the proliferation of A549 cells in a dose-dependent manner. (**C**) Gm15290 knockdown promoted the apoptosis of A549 cells in a dose-dependent manner. (**D**) Gm15290 knockdown reduced the invasion of A549 cells in a dose-dependent manner. The Gm15290 siRNA at concentrations of 20, 40, and 80 nM were respectively transfected into A549 NSCLC cells. After incubation for 48 h, the Gm15290 enrichment, cell proliferation, cell apoptosis, and cell invasion were detected. *P<0.05 compared with scrambled siRNA (scramble).

### Gm15290 directly interacted with *miR-615-5p*, and its levels in NSCLC patients were inversely correlated with the levels of the tumor suppressor *miR-615-5p*

To explore the underlying mechanism of Gm15290 promoting the NSCLC cell proliferation and invasion, we searched the potential RNA targets of Gm15290. The output of RNA hybrid online server showed that Gm15290 potentially targetted the tumor suppressor *miR-615-5p* (Figure 4A). The analysis on *miR-615-5p* expression in the cell lines displayed that, compared with HBE cells, *miR-615-5p* was dramatically decreased in NSCLC cell lines SK-MES-1, A549, and NCI-H460 (Figure 4B). Pearson correlation coefficient analysis showed that the levels of Gm15290 were inversely correlated with *miR-615-5p* levels in NSCLC patients (Figure 4C). Then, RNA pull-down assays were used to validate the interaction of Gm15290 with *miR-615-5p* mutually. In the RNA complex pulled down by the biotinylated DNA probe complementary to Gm15290, a fairly high level of *miR-615-5p* was detected (Figure 4D). Furthermore, in the RNA complex pulled down by the biotinylated probe complementary to *miR-615-5p*, a relatively high level of Gm15290 was detected (Figure 4E). These data demonstrate that Gm15290 can directly interact with *miR-615-5p* and suggest that the role of Gm15290 in NSCLC cell proliferation and invasion may be associated with *miR-615-5p*.

The article "lncRNA Gm15290 promotes cell proliferation and invasion in lung cancer through directly interacting with and suppressing the tumor suppressor miR-615-5p" was published in 2018. Journal: Biosci Rep.

**Figure 4:** lncRNA Gm15290 directly targetted *miR-615-5p*, and Gm15290 levels were inversely correlated with *miR-615-5p* levels in NSCLC patients (**A**) Details of the binding potential between Gm15290 and *miR-615-5p* evaluated by the RNA hybrid bioinformatic tool. (**B**) *miR-615-5p* was sharply decreased in NSCLC cell lines. (**C**) Pearson correlation coefficient analysis for the correlation between Gm15290 and *miR-615-5p* levels in 30 NSCLC patients. (**D**) RNA pull-down assay for the binding of Gm15290 and *miR-615-5p* using Gm15290 cDNA probe. Biotinylated Gm15290 cDNA probe was applied to pull down the Gm15290/*miR-615-5p* RNA complex, and the level of *miR-615-5p* in the complex was detected with Northern blotting. NB represents Northern blotting. (**E**) RNA pull-down assay for the binding of Gm15290 and *miR-615-5p* using *miR-615-5p* cDNA probe. Biotinylated *miR-615-5p* cDNA probe was applied to pull down the Gm15290/*miR-615-5p* RNA complex, and the Gm15290 enrichment in the complex was detected with qPCR. Input: 20% of total RNA, regarded as a positive control. Control probe: a scrambled probe was used as a negative control. **P<0.01.

### Gm15290 suppressed *miR-615-5p* expression, and its promotion on A549 cell proliferation and invasion could be antagonized by *miR-615-5p*

To confirm that the role of Gm15290 in NSCLC cell proliferation and invasion is associated with *miR-615-5p*, the effect of Gm15290 on the expression of *miR-615-5p* and its target genes were investigated. Overexpression of Gm15290 sharply reduced the level of *miR-615-5p*, and knockdown of Gm15290 distinctly increased *miR-615-5p* expression in A549 cells (Figure 5A). As expected, Gm15290 overexpression promoted and Gm15290 knockdown suppressed the expression of *miR-615-5p* target genes, including *IGF2, AKT2*, and *SHMT2* that are all proto-oncogenes (Figure 5B). Finally, Gm15290 and *miR-615-5p* were individually or jointly overexpressed in A549 cells. Our results showed that *miR-615-5p* antagonized the promotion of Gm15290 on A549 cell proliferation and invasion (Figure 5C,E). Simultaneously, *miR-615-5p* rescued the suppression of Gm15290 on A549 cell apoptosis (Figure 5D). These results indicate that Gm15290 promotes A549 cell proliferation and invasion through suppressing the tumor suppressor *miR-615-5p*.

The article "lncRNA Gm15290 promotes cell proliferation and invasion in lung cancer through directly interacting with and suppressing the tumor suppressor miR-615-5p" was published in 2018. Journal: Biosci Rep.

**Figure 5:** Gm15290 negatively regulated *miR-615-5p* expression, and its promotion on A549 cell proliferation and invasion was antagonized by *miR-615-5p* (**A**) Gm15290 negatively regulated *miR-615-5p* expression. (**B**) Gm15290 positively regulated expression of *miR-615-5p* target genes *IGF2, AKT2*, and *SHMT2*. IGF2: insulin-like growth factor 2; AKT2: serine/threonine kinase; SHMT2: serine hydroxymethyltransferase 2. To investigate the role of Gm15290 in *miR-615-5p* expression, 2 μg/ml pcDNA-Gm15290, and 40 nM Gm15290 siRNA were respectively transfected into A549 cells. After incubation for 48 h, expression of *miR-615-5p* was detected with qPCR and the protein levels of *IGF2, AKT2*, and *SHMT2C* were detected with Western blotting. (**C**) *miR-615-5p* antagonized the promotion of Gm15290 on A549 cell proliferation. (**D**) *miR-615-5p* rescued the suppression of Gm15290 on A549 cell apoptosis. (**E**) *miR-615-5p* antagonized the promotion of Gm15290 on A549 cell invasion. Total of 2 μg/ml of pcDNA-Gm15290 and 60 nM of miR-615-5p mimic were individually transfected or co-transfected into A549 cells. After incubation for 48 h, cell proliferation, apoptosis, and invasion were detected. **P<0.01.

## Discussion

lncRNA Gm15290 was discovered by mRNA expression profiling in the brain of mice with hereditary catalepsy in 2014 [25]. During the past 3 years, there have been rare reports that reveal the exact functions of Gm15290 in any biological processes. Recently, an integrated analysis for transcription factors, miRNAs and lncRNAs revealed that Gm15290 was up-regulated in animals with obliterative bronchiolitis [26]. This integrated analysis indicates that Gm15290 was expressed in the lung and suggests that Gm15290 might play a role in the progression of lung diseases. In the present study, we found that Gm15290 was significantly up-regulated in human NSCLC tissues and NSCLC cell lines, compared with the adjacent normal tissues and HBE normal lung epithelial cell line. Then, our data on gain- and loss-of-function experiments demonstrated that Gm15290 positively regulated the proliferation and invasion of NSCLC cells.

The interaction between different categories of ncRNAs and their interaction with protein coding genes play important roles in tumor occurrence and development [27]. Competing endogenous RNA (ceRNA) is a quite famous hypothesis that reveals a typical mechanism for the interaction between RNAs [28]. As known, a miRNA directly targets the mRNA of a specific gene (called the target gene of a miRNA) to inhibit the expression of its protein. A ceRNA molecule (usually a lncRNA or a circular RNA) can regulate the expression of the target gene by competitive binding to their shared miRNA. In this mechanism, lncRNAs bind to specific miRNAs, decrease their levels, and alleviate their inhibitory effect on the target genes [28,29]. It has been revealed that some lncRNAs directly interacted with tumor promoting or tumor suppressor miRNAs in NSCLC [30,31]. For instance, lncRNA urothelial carcinoma-associated 1 (UCA1) overexpression enhanced, whereas UCA1 knockdown impaired the proliferation and colony formation of NSCLC cells; UCA1 targetted and suppressed the *miR-193a-3p* level, and promoted the expression of human epidermal growth factor receptor 4, an identified target gene of *miR-193a-3p* [22]. Another example is that lncRNA H19 targets and down-regulates *miR-107*, and promotes cell cycle progression of NSCLC cells [32]. In the present study, we found that Gm15290 overexpression suppressed, whereas Gm15290 knockdown increased the level of *miR-615-5p* in A549 NSCLC cells. Our data on RNA pull-down assays revealed that Gm15290 could directly target *miR-615-5p*. Furthermore, Gm15290 positively regulated the expression of *miR-615-5p* target genes *IGF2, AKT2*, and *SHMT2*.

The article "lncRNA Gm15290 promotes cell proliferation and invasion in lung cancer through directly interacting with and suppressing the tumor suppressor miR-615-5p" was published in 2018. Journal: Biosci Rep.

In pancreatic ductal adenocarcinoma, *miR-615-5p* targetted AKT2 and inhibited AKT2-mediated cell proliferation [33]. In hepatocellular carcinoma, *miR-615-5p* was able to target *IGF2* and *SHMT2* and inhibited cell proliferation, invasion, and metastasis [34,35]. However, the exact role of *miR-615-5p* in the progression of NSCLC has not been reported. In the present study, we showed that overexpression of *miR-615-5p*, by the *miR-615-5p* mimic transfection, significantly suppressed A549 cell proliferation and invasion, and markedly promoted cell apoptosis. Furthermore, *miR-615-5p* could antagonize the promotion of Gm15290 on A549 cell proliferation and invasion and rescue the suppression of Gm15290 on A549 cell apoptosis, indicating that Gm15290 promotes A549 cell proliferation and invasion through suppressing *miR-615-5p*. Similar to the results of our study, a quite recent miRNA profiling assay in patients with lung cancer revealed that *miR-615-5p* was positively correlated with survival in stage I lung cancer [36].

In conclusion, lncRNA Gm15290 might function as a tumor promoting gene in NSCLC. It promotes cell proliferation and invasion in NSCLC through directly targetting and suppressing the tumor suppressor *miR-615-5p*.

## Abbreviations

ceRNA: competing endogenous RNA
EDTA: ethylenediaminetetraacetic acid
HOTAIR: HOX transcript antisense RNA
lncRNA: long non-coding RNA
NSCLC: non-small cell lung cancer
PVDF: polyvinylidene fluoride
UCA1: urothelial carcinoma-associated 1
